The article "Detection of ESBL among ampc producing enterobacteriaceae using inhibitor-based method" was retracted in 2014. Reason: plagiarism.

# Detection of ESBL among ampc producing enterobacteriaceae using inhibitor-based method

**DOI:** 10.11604/pamj.2013.14.28.1347

**Published:** 2013-01-20

**Authors:** Sasirekha Bakthavatchalu, Uma Shakthivel, Tannu Mishra

**Affiliations:** 1 Department of Microbiology, Centre for Post Graduate Studies, Jain University, Bangalore, Karnataka- 560 011, India

**Keywords:** boronic acid, ESBL, ampc beta-lactamases, enterobacteriaceae, cefepime

## Abstract

**Introduction:**

The occurrence of multiple β-lactamases among bacteria only limits the therapeutic options but also poses a challenge. A study using boronic acid (BA), an AmpC enzyme inhibitor, was designed to detect the combined expression of AmpC β-lactamases and extended-spectrum β-lactamases (ESBLs) in bacterial isolates further different phenotypic methods are compared to detect ESBL and AmpC.

**Methods:**

A total of 259 clinical isolates of *Enterobacteriaceae* were isolated and screened for ESBL production by (i) CLSI double-disk diffusion method (ii) cefepime- clavulanic acid method (iii) boronic disk potentiation method. AmpC production was detected using cefoxitin alone and in combination with boronic acid and confirmation was done by three dimensional disk methods. Isolates were also subjected to detailed antibiotic susceptibility test.

**Results:**

Among 259 isolates, 20.46% were coproducers of ESBL and AmpC, 26.45% were ESBL and 5.40% were AmpC. All of the 53 AmpC and ESBL coproducers were accurately detected by boronic acid disk potentiation method.

**Conclusion:**

The BA disk test using Clinical and Laboratory Standards Institute methodology is simple and very efficient method that accurately detects the isolates that harbor both AmpCs and ESBLs.

## Introduction

The rapid global dissemination of *Enterobacteriaceae* harboring plasmid-borne extended-spectrum β-lactamases (ESBLs) and plasmid-mediated AmpC β-lactamases represents a significant clinical threat [1, 2]. ESBLs producing organism confer resistance to penicillin, cephalosporins, and monobactams. They cannot hydrolyze cephamycins and are inhibited by clavulanic acid (CA) [3]. Like ESBLs, plasmid-mediated AmpC β-lactamases have a broad substrate profile that includes penicillin, cephalosporins, and monobactams. In contrast to ESBLs, they hydrolyze cephamycins and are not inhibited by commercially available β-lactamase inhibitors [4, 5]. Inappropriate use of cephalosporins in clinical practice led to the emergence of bacteria producing multiple β-lactamases. This leads to therapeutic failure when β-lactam drugs or β-lactam/inhibitor combination are used [6].

The ESBL confirmation methods have been established by Clinical Laboratory Standards Institute (CLSI) and are used worldwide [7]. Currently there are no CLSI recommended guidelines to detect AmpC β-lactamases. Several methods of phenotypic detection of AmpC β-lactamases are described; however, these methods are labor intensive and subjective, lack sensitivity and/or specificity and cannot be adopted on a routine basis. PCR gives satisfactory results, but it is costlier and time consuming, and equipment availability is limited to few laboratories [8–15].

The CLSI recommended phenotypic confirmatory test would fail to detect ESBL in the presence of AmpC, as the latter enzyme is resistant to clavulanic acid [10]. Clavulanic acid induces high level expression of chromosomal AmpC β-lactamases, masking the synergy arising from the inhibition of an ESBL. Thus, the coexistence of both ESBL and AmpC β-lactamases in the same strain may result in false-negative tests for the detection of ESBLs [16].

Boronic acid (BA) derivatives were reported as reversible inhibitors of AmpC enzymes [17, 18]. Several studies have validated the use of boronic acid to detect AmpC β-lactamases among Gram-negative bacteria [16, 19–21]. Rapid and accurate detection of ESBLs and AmpC β-lactamases is important to guide proper antimicrobial therapy and for appropriate infection control measures. Therefore the present study was aimed to evaluate the usage of boronic acid in a phenotypic confirmatory test to detect ESBL among AmpC β-lactamases producing isolates.

## Methods

### Bacterial isolates

A total of 259 consecutive nonrepetitive clinical isolates of *Enterobacteriaceae* were isolated from various clinical samples such as urine (*n*= 103), pus (*n*=83), sputum (*n*= 60), blood (*n*= 9) over a period of six months from January 2010 to June 2010. Samples were processed and isolates were identified on the basis of conventional microbiological procedures [22].

### Antimicrobial susceptibility testing

Antibiotic susceptibility was determined by Kirby- Bauer disk diffusion method and the results were interpreted according to the guidelines of the Clinical Laboratory Standard Institute [23]. The antibiotics used were ampicillin (10µg), ticarcillin(75µg), piperacillin(100µg), amoxycillin/ clavulanic acid (20/10µg), ticarcillin/clavulanic acid (75/10µg), piperacillin- tazobactum (100/10µg), aztreonam (30µg), cephotaxime (30µg), ceftazidime(30µg), ceftriaxone (30µg), cefepime (30µg), impenem (10µg), gentamicin (10µg), amikacin (30µg), tetracycline (30µg) and ciprofloxacin (5µg), chloramphenicol (30µg). *E. coli* ATCC 25922 was used as a quality control strain.

All the 259 isolates were screened for ESBL production by (i) CLSI double-disk diffusion method [23] (ii) cefepime- clavulanic acid method (iii) boronic disk potentiation method. AmpC production was detected using cefoxitin alone and in combination with boronic acid and confirmation was done by three dimensional disk method. Briefly, 5µl of the freshly prepared clavulanic acid (2g/l of PBS at pH 6) was added to cefotaxime (30µg; CTX+CA) and cefepime (30µg; CPM+CA) disks. Then 5 µl of 3- amino phenyl boronic acid (Sigma Aldrich, India) stock solution (60g/l of DMSO) was added to cefotaxime disc with(CTX+CA+BA) and without clavulanic acid(CTX+BA) and also to cefoxitin disc(FOX+BA). The discs were placed onto Mueller hinton agar plates containing lawn culture of 0.5 McFarland unit of test organism. The plates were incubated at 37° C for 18-24 hrs. The results were interpreted as follows:

1. A ≥ 5 mm increase in the zone diameter of the cefotaxime alone (CTX) and in combination with clavulanic acid (CTX+CA) or boronic acid (CTX+BA) was indicative of ESBL or AmpC production
2. A ≥ 5 mm increase in the zone diameter of CTX+BA and CTX+CA versus CTX+CA+BA was indicative of combined ESBL and AmpC production
3. A ≥ 5 mm increase in the zone diameter of the CPM alone and in combination with clavulanic acid (CPM+CA) was indicative of ESBL production
4. A ≥ 5 mm increase in the zone diameter of the Cefoxitin (FOX) alone and in combination with boronic acid (FOX+BA) was considered positive for AmpC production

All 259 isolates were subjected to a modified three dimensional extract test to confirm AmpC production [23].

## Results

Of the total 259 *Enterobacteriaceae* isolates, 115 were *Escherichia coli* (44.4%), 59 (22.77%) were *Klebsiella pneumonia*, 41 (15.83%) were *Proteus mirabilis*, 29(11%) were *Enterobacter cloacae*, and 15 *Citrobacter* spp. Among 259 clinical isolates of *Enterobacteriaceae*, 68 (26.25%) and 14(5.4%) were pure ESBL and AmpC producers respectively; 53 (20.46%) isolates were combined ESBL and AmpC producers; and 124 (47.87%) of the isolates did not harbor any type of enzyme (Table 1). In our study the prevalence of ESBL and AmpC co- producing isolates was 20.46%, which is relatively low (27.5% and 33.7%) compared to the previous report [25, 26]. This variation may be due to different pattern of antibiotic use and differences in the study group.

**Table 1:** Extended-spectrum beta-lactamases and AmpC producing *Enterobacteriaceae*

Organisms	Pure ESBL (%)	Pure AmpC	ESBL+ AmpC	Negative	Total
*E coli*	30 (26)	3 (2.60)	18 (15.65)	64 (55.65)	115
*K pneumoniae*	19 (32.20)	4 (6.77)	21 (35.59)	15 (25.42)	59
*E cloacae*	5 (12.19)	3 (7.31)	6 (14.63)	27 (65.85)	41
*P mirabilis*	11(37.93)	2(6.89)	5 (17.24)	11(37.93)	29
*Citrobacter* spp	3 (20)	2 (13.33)	3 (20)	7 (46.66)	15
**Total**	**68 (26.25)**	**14 (5.40)**	**53 (20.46)**	**124 (47.87)**	**259**

ESBL: Extended-spectrum beta-lactamases

CLSI double-disk diffusion method detected all ESBL producers (100%) but in combined ESBL and AmpC failed to detect 16 (30.18%), ESBL producers. The average increases in the zone diameters of the CTX discs in the presence of either CA and BA was 14.1 mm and 13.2 mm respectively were higher than those for the CLSI confirmatory test 11.3 mm and 10.9 mm, respectively. The rate of detection of ESBLs by the CLSI confirmatory test for clinical isolates that produce both ESBLs and AmpC (20.46%) was lower than that for clinical isolates that produce ESBLs but not AmpC (26.45%). If CLSI double-disk diffusion method was used alone, 6% of ESBL producing organisms would have been missed. The average increases in the zone diameters of the CTX disc in the presence of both CA and BA was 10.7 mm and 8.3 mm, which is higher than that of CLSI confirmatory test 7.1 mm and 5.1 mm, respectively. CLSI double-disk diffusion method was able to detect only 105 of 121 ESBL producing isolates but it detected all ESBL negative isolates correctly. Sturenburg *et al* [27] reported that the cefepime-clavulanic acid (CPM-CA) method could reliably detect ESBL in the presence of AmpC, in our study CPM+CA potentiated disc detected all ESBL producers whether alone or in combination with AmpC correctly (Table 2).

**Table 2:** Comparison of phenotypic method with boronic acid disk potentiation method for extended-spectrum beta-lactamases detection

Phenotypes	CLSI double-disk diffusion method	CTX+BA for AmpC	CTX +CA+BA for ESBL + AmpC	CPM + CA for ESBL	
				Positive	Negative
Pure ESBL (*n*= 68)	68	0	68	68	0
Pure AmpC (*n*= 14)	0	14	14	0	14
ESBL + AmpC (*n*= 53)	37	43	53	53	0
Negative (*n*=124)	0	0	0	0	124
Total (*n*= 259)	105	57	135	121	138

CLSI: Clinical Laboratory Standards Institute; CTX+CA+BA: Cefotaxime disc with clavulanic acid; CTX+BA: Cefotaxime disc without clavulanic acid; ESBL: Extended-spectrum beta-lactamases; CPM-CA: Cefepime-clavulanic acid

## Discussion

The occurrence of multiple β-lactamases among bacteria only limits the therapeutic options but also poses a challenge for microbiology laboratories to identify them [6]. The detection of the co-production of ESBL and AmpC is essential for enhanced infection control and effective anti-microbial therapy. There is no CLSI described guidelines for the detection of multiple β-lactamases. There is a paucity of data from Indian laboratories on the coexistence of multiple beta lactamases in individual isolates. Possible approaches to overcome this difficulty of ESBL detection in the presence of AmpC include the use of tazobactam or sulbactam, which are much less likely to induce AmpC β-lactamases or preferable use of inhibitors to ESBL detection tests [24].

All AmpC enzymes can hydrolyze cephamycins except ACC-1, which makes this drug better screening agents for AmpC production [28]. In the present study cefoxitin resistance was seen in 86/259 (33.20%) isolates. All the 67 (100%) AmpC producing isolates (100%) showed resistance to cefoxitin disc, but only 62/67 (93%) showed ≥ 5mm zone diameter with FOX+BA discs. None of the cefoxitin sensitive isolates showed AmpC production. The isolate which does not harbor AmpC, zone sizes of disks containing FOX and FOX+BA were the same. Modified three dimensional extract method detected 61 isolates (91%) as AmpC producers. All the negatives were identified correctly (Table 3). FOX resistance in isolates that did not show any enhancement with the addition of BA, resistance may be due other mechanisms like porin channel alterations in these isolates. Our study correlated with that of Song *et a*l. [20] who showed 97.7% sensitive for AmpC detection by FOX-BA method, where our study showed 91% sensitivity. Pure AmpC β-lactamases were detected only in 5.40% of the isolates. This prevalence was lower than compared to the reports from other parts of the world [12, 29]. Two Indian studies reported 8 and 43% prevalence of AmpC β-lactamases [15, 30]. In all these AmpC producers, we were not able to distinguish between the chromosomal derepressed and plasmid mediated enzymes as this requires genotypic confirmatory tests.

**Table 3:** Occurrence of cefoxitin resistance and efficacy of FOX-BA disk test for detection of AmpC among Enterobacteriaceae

Phenotypes	FOX (Cefoxitin disk resistance)		FOX+BA disc for AmpC		
	R (%)	S (%)	≥5mm enhancement	FOX disc resistant, no zone enhancement	FOX disc senstitive, no zone enhancement
Pure ESBL (*n*= 68)	19	49	0	19	49
Pure AmpC (*n*= 14)	14	0	12	2	0
ESBL+AmpC (*n*= 53)	53	0	50	3	0
Negative (*n*=124)	0	124	0	0	124
Total (*n*= 259)	86 (33)	173 (67.79)	62(23.93)	24(9.26)	173(66.79)

ESBL: Extended-spectrum beta-lactamases

In our study ESBL and AmpC co producing isolates were predominantly from K. *pneumonia* (35.59%) followed by E. *coli* (15.65%). Isolates producing both ESBL and AmpC showed greater resistance to most of the antibiotics. Greater resistance to β-lactam and non β-lactam antibiotics was evident in isolates coproducing both ESBL and AmpC producers than in pure ESBL/AmpC isolates. Combination of β-lactam/ β-lactam inhibitor showed greater activity in both groups, this is likely to be due to the heavy selection pressure from overuse of these antibiotics and seem to be losing the battle [31]. Piperacillin/ tazobactum showed less resistance as compared to ticarcillin/ clavulanic acid and amoxycillin/ clavulanic acid. Among aminoglycosides, amikacin showed grater activity against all the isolates irrespective of their resistance status (Table 4). Sensitivity to imipenem was observed to be 100%, which is in concordance with the studies conducted by other workers. Sensitivity to imipenem, which again advocates the usage of carbapenem antibiotics as the therapeutic alternative to β-lactam antibiotics as indicated in many studies [32, 33].

**Table 4:** Comparison of antimicrobial resistance patterns of isolates harboring both extended-spectrum beta-lactamases and AmpC

Antimicrobials	Resistant pattern of ESBL and AmpC producer (*n =*53) % Resistant
Ampicilin	97.95
Ticarcillin	95.91
Piperacillin	81.63
Amoxycillin/clavulanic acid	42.85
Ticarcillin/clavulanic acid	73.46
Piperacillin- tazobactum	36.73
Aztreonam	83.67
Cephotaxime	85.71
Ceftazidime	81.63
Ceftriaxone	83.67
Cefepime	63.26
Impenem	0
Gentamicin	69.38
Amikacin	73.46
Tetracycline	65.30
Ciprofloxacin	53.06
Chloramphenicol	48.97

ESBL: extended-spectrum beta-lactamases

## Conclusion

A mixed type of drug resistance mechanisms seem to operate in the isolates tested. The results of the study indicate that the current CLSI recommended methods to confirm ESBL enzymes by conducting clavulanate synergy tests with ceftazidime and cefotaxime may be insufficient for ESBL detection in clinical isolates of *Enterobacteriaceae* since these organisms often produce multiple β-lactamses. Inhibitor based method using boronic acid disc test, practical and efficient method that uses current CLSI methodology to detect co- producing ESBL and AmpC β-lactamase is a suitable alternative to test ESBL.
